This article has been retracted.

# Grading Evaluation of Cardiotoxicity in Patients with Breast Cancer Treated with Adjuvant Paclitaxel Anthracycline/Cyclophosphamide Chemotherapy: A Meta-Analysis

**DOI:** 10.1155/2022/7963146

**Published:** 2022-08-08

**Authors:** Weibao Hu, Mengli Song, Linfeng Li

**Affiliations:** ^1^Department of Cardiology, The Fifth People's Hospital of Shangrao City, Jiangxi Province, Shangrao 334099, China; ^2^Jiangxi Provincial People's Hospital Affiliated to Nanchang University, Nanchang 330006, China; ^3^Department of Cardiology, Jiangxi Provincial People's Hospital, Nanchang 330006, China

## Abstract

**Objective:**

The cardiac safety of concurrent treatment with anthracycline (A), cyclophosphamide (C), and paclitaxel (T) in an adjuvant BC treatment regimen is still under debate. In this study, we aimed to determine cardiotoxicity events following ACT chemotherapy among operable breast cancer patients without HER2-positive.

**Methods:**

We searched PubMed and the Cochrane Library for RCTs prior to July 2019 evaluating the cardiac impairment of ACT chemotherapy regimens in BC patients. The search terms were “BC,” “chemotherapy,” “docetaxel or “doxorubicin,” “paclitaxel,” and “cyclophosphamide.” Cardiotoxic events included LVEF decline ≥ 10 points, congestive heart failure (CHF), and cardiac death.

**Results:**

In total, 12 studies with 4032 subjects were included in this meta-analysis, and all patients received ACT regimen. The analysis results indicated that LVEF decrease ≥ 10 points was the most common cardiotoxic event (16%; (95% CI (8%–24%)) with *χ*^2^ = 95.75, *P* < 0.001, *I*^2^ = 95.8%). CHF showed the lowest rate (1%; (95% CI (0%–1%)) with *χ*^2^ = 8.00, *P* = 0.433, *I*^2^ = 0.0%). Subgroup analysis demonstrated that the incidence of CHF due to A → C → T chemotherapy regimen was lower than that of other events, however, without significance. No significant difference was observed in the occurrence of cardiac death.

**Conclusion:**

The ACT regimen in patients with HER2-negative BC was associated with an increased risk of adverse cardiactoxic events.

## 1. Introduction

Breast cancer (BC) is a common female malignant tumor, and its incidence is increasing year by year. In cities with high stress levels, the incidence rate of BC is the highest among all female malignant tumors [1]. Chemotherapy can provide long-term relief from breast cancer pain and improve patient survival. Therefore, treatment with adjuvant chemotherapy after breast cancer surgery is recommended. The most commonly used chemotherapy drugs included anthracycline, cyclophosphamide, and paclitaxel. ACT which is composed of anthracycline, cyclophosphamide, and paclitaxel is a most commonly used chemotherapy regimen. Anthracycline has been evaluated as the most effective drug for chemotherapy, and it is extensively used in the treatment of solid tumors and leukemia in adults and children [2]. Nevertheless, the application of ACT is limited because of evident cardiotoxicity during anthracycline treatment. Cardiotoxicity from anthracyclines is progressive and irreversible and may cause cardiotoxicity even at low doses. Impaired left ventricular ejection fraction (LVEF) and chronic heart failure (HF) with anthracycline regimens compared to nonanthracycline regimens were 5 times higher than nonanthracycline regimens [3, 4]. Risk of cardiotoxicity associated with lifetime cumulative exposure to anthracyclines [5]. Paclitaxel, a semisynthetic plant anticancer drug, showed definite anticancer effects in the BC treatment. Its risk for cardiac toxicity is unknown, and only few studies have reported paclitaxel-related cardiac events, including asymptomatic ECG abnormalities, arrhythmia, and myocardial infarction [6, 7]. Cyclophosphamide is the cornerstone of adjuvant and metastatic BC; it is also used in the treatment of majority of early and advanced diseases [8]. Combination therapy can reduce the toxic accumulation of chemotherapeutic drugs more markedly than monotherapy. The cardiotoxicity of anthracycline, cyclophosphamide, and paclitaxel has been evaluated only when administered alone [9–12]. We first evaluate the cardiotoxicity of combined chemotherapy in breast cancer patients. Antitumor drug cardiotoxicity refers to toxic effects on the myocardial or cardiac electrical conduction system in cancer patients after treatment with certain antitumor drugs, resulting in heart disease [13]. HF risk after antineoplastic drug treatment remains a lifelong threat, particularly in young women with longer life expectancy after successful cancer treatment [14, 15]. However, in practical clinical applications, chemotherapy drugs for breast cancer are often used in combination. With this rationale, we conducted this meta-analysis to obtain an overall understanding of cardiotoxicity caused by ACT chemotherapy.

## 2. Patients and Methods

### 2.1. Identification of Trials

According to PRISMA, we performed a meta-analysis of randomized controlled trials (RCTs) by seeking the Web Scientific and PubMed databases. This meta-analysis includes RCTs published prior to July 2019 evaluating the cardiac damage of CAP chemotherapy regimens in BC patients [16]. The search terms were used: “BC,” “chemotherapy,” “docetaxel or “doxorubicin,” “paclitaxel,” and “cyclophosphamide.” Manual and independent searches of reference lists of eligible articles for additional sources. No language restriction was applied.

### 2.2. Selection Criteria

Two authors (HT and BYX) independently performed an initial search, deduplicated records, screened records by title and abstract, and identified records by scanning the full text of publications. The study inclusion criteria are as follows: (1) type of study, phase III RCT; (2) the subjects were women aged 18 years and older with a pathological diagnosis of BC; (3) sufficient data were available, including regimen, observation period, and number of outcome events; and (4) outcome indicators, (i) cardiac events including LVEF decrease ≥10 points, (ii) severe cardiac events including CHF, and (iii) cardiac death [7, 8]. The exclusion criteria were as follows: (1) information not sufficient to extract literature for data analysis and (2) trials of HER2 inhibitor-containing regimens.

### 2.3. Data Extraction

Experimental data were extracted independently from eligible studies by two researchers. Basic characteristics of the study were further extracted, including year of publication, ethnicity, country of origin, the first author's last name, and study design. The collected data are presented in Table 1. Article authors were contacted for missing data; any discrepancies were resolved by discussion with other authors.

### 2.4. Risk of Bias Assessment

Individual studies were assessed for risk of bias using Review Manager 5.3 from the Cochrane Collaboration. Our meta-analysis used the Cochrane Consensus-recommended harmonized criteria including the following six items: selection bias, performance bias, detection bias, attrition bias, reporting bias, and other potential biases used previously.

### 2.5. Quality Assessment

The quality of each included study was assessed using the Quality Assessment of Studies for Diagnostic Accuracy (QUADAS-2).

### 2.6. Statistical Analysis

Statistical analysis was performed using Stata 12.0 software. Spearman's correlation coefficients for log sensitivity and 1-specificity were calculated to detect threshold effects. *χ*^2^ Cochran's *Q* test and Higgins's *I*^2^ statistic were used to assess heterogeneity between studies. Heterogeneity between studies was assessed by using *χ*^2^ Cochran's *Q* test and Higgins's *I*^2^. An *χ*^2^ = 95.75, *P* < 0.001, *I*^2^ = 95.8% was considered significant heterogeneity. Pooled rates of cardiac events were calculated using bivariate random-effects regression models with 95% confidence intervals (CIs). In addition, Fagan's nomogram formula is also used. Finally, publication bias was assessed using Deeks's funnel plot asymmetry test. All *P* values are two-sided.

## 3. Results

### 3.1. Data Selection

In the initial search, a total of 424 records were affirmed through systematic searches and human review. After removing duplicate records, there were a total of 296 abstracts. After an initial review of titles and abstracts, we excluded 238 records, of which 58 articles were considered potentially eligible for inclusion. In addition, we excluded 16 records for the following reasons: studies not related to cardiotoxicity or to the ACT regimen (4 cases) and insufficient data (12 cases). Finally, a total of 12 articles were included in the meta-analysis (Figure 1).

### 3.2. Study Characteristics and Quality Assessment

The 12 selected publications were published from 1997 to 2017 and described twelve studies comprising 4032 patients with BC. All studies were written in English. The included articles' quality was evaluated by calculating the QUADAS-2 score (Figure 2). Most trials were anthracycline+cyclophosphamide+paclitaxel regimen sequence, while one trial was paclitaxel+anthracycline+cyclophosphamide regimen sequence. All the included studies had QUADAS-2 scores > 8, which indicated a high quality.

### 3.3. Meta-Analysis

The results confirmed that there was heterogeneity in our meta-analysis (*χ*^2^ = 11.255, *P* = 0.002; *I*^2^ = 82.23%). Consequently, this study chose the random effects model. The overall incidence of cardiac toxicity events was 6.5% (*n* = 262; 95% CI), indicating a low occurrence of cardiotoxicity due to ACT regimens in adjuvant treatment. LVEF decrease ≥10 points was the most frequently occurring cardiac toxicity (16%; 95% CI (8%–24%)) with *χ*^2^ = 95.75, *P* < 0.001, *I*^2^ = 95.8% (Figure 3). Incidence of congestive HF was (1%; 95% CI (0%–1%)) with *χ*^2^ = 8.00, *P* = 0.433, *I*^2^ = 0.0% (Figure 4). However, the incidence of cardiac death was 0% (Figure 5). We further performed subgroup analyses according to different treatment regimens. The incidence rate of LVEF decrease ≥10 points in both A ⟶ C ⟶ T regimen sequence and other regimen sequence was identical (16%) (Figure 6). The incidence of congestive HF was 1% in A → C → T regimen sequence and 2% in others (A ⟶ T ⟶ C and T ⟶ A + C) (Figure 7). The heterogeneity between the two groups was 0.316, suggesting a difference in the incidence of congestive HF in different protocol sequences.

### 3.4. Publication Bias

To investigate potential publication bias, we performed Deeks' funnel plot asymmetry test (Figures 8 and 9). The resulting *P* value indicates the absence of publication bias in the subgroup analysis.

## 4. Discussion

We performed a meta-analysis to determine the occurrence of cardiotoxicity following the ACT regimen in BC patients in this study. We discovered that the ACT regimen was associated with an increased risk of adverse cardiac events.

A growing number of studies describe the incidence of cardiotoxicity, including congestive heart failure, decreased LVEF, and/or cardiac death, in BC patients treated with CAP regimens [5, 6]. However, there is still a lack of systematic statistical analysis to evaluate the occurrence of cardiotoxicity. Therefore, we included 12 articles published between 1997and 2017 involving 12 independent studies comprising 4032 patients with BC to perform a detailed meta-analysis about the toxicity of ACT regimen. This page is the first meta-analysis to assess the cardiotoxicity of paclitaxel+anthracycline+cyclophosphamide regimen in BC patients. Currently, combination chemotherapy with paclitaxel, anthracyclines, and cyclophosphamide is an important treatment option for BC. Some studies have reported that combination chemotherapy can reduce the cardiotoxicity of each chemotherapy drug to a certain extent [16–18]. However, some studies demonstrated that concurrent usage of adriamycin and paclitaxel would increase cardiotoxicity, because taxanes would change metabolism process of adriamycin and increase its serum drug concentration [19]. We evaluated the effects of different regimen sequences based on different cardiotoxicity grades. Our findings showed that the most common cardiotoxicity was LVEF decrease (16%). Congestive HF and cardiac death were rare (1% and 0%, respectively). Subgroup analysis indicated an insignificant occurrence of cardiac toxicity events in other regimen sequences. Therefore, our results had confirmed that ACT regimens was associated with increased cardiotoxicity.

Since heart injury such as reduced cardiofunction would impact subsequent treatment, especially among elderly or patients with cardiocerebral vascular disease, physician shall take both excellent efficacy and obvious cardiotoxicity of ACT in consideration when choosing ACT regimen and take measures to avoid or reduce chemotherapy drug-related cardiotoxicity, such as reducing dosage and using different forms, different combinations, and cardioprotector.

This study has several limitations. First, the quality in determining cardiac outcomes is affected by sample size variability and underreporting, which may not be sufficient to accurately estimate rare outcomes. Second, in some studies, they were reported only in specific subsets of participants. Third, the doses of chemotherapeutics we included were not uniform. Due to the unique therapeutic concentrations of these drugs, it is difficult to assess their unit cardiotoxicity. Fourth, publication bias analysis suggests potential publication bias. Therefore, high-quality and more large-scale clinical studies are needed to supplement and validate our results. This study included in this meta-analysis were conducted in various ethnic groups and countries. The differences in ethnic groups and those in the development of medical standards are likely to lead to the emergence of heterogeneity.

## 5. Conclusion

The ACT regimen may be a relatively safe treatment regimen for BC in terms of cardiotoxicity and efficacy. The results of our meta-analysis provide a new reference for clinical strategies using the ACT regimen for BC.

## Figures and Tables

**Figure 1:** Flow diagram and results of literature screening.

**Figure 2:** Quality assessment and bias risk assessment in the study included in the meta-analysis.

**Figure 3:** The overall incidence of LVEF decrease ≥10 points.

**Figure 4:** The overall incidence of congestive heart failure.

**Figure 5:** The overall incidence of congestive cardiac death.

**Figure 6:** Incidence of LVEF decrease ≥10 points in the A → C → T regimen sequence group and the other group.

**Figure 7:** Incidence of congestive heart failure in the A → C → T regime sequence group and the other group.

**Figure 8:** Funnel plot of LVEF decrease ≥10 points.

**Figure 9:** Funnel plot of congestive heart failure.

**Table 1:** Characteristics of study included in the meta-analysis.

Author	Published year	Country	Regimes sequence	Age median	Observation period	Setting	Cardiac toxicities
Dennis J Slamon	2011	USA	A+C→T(N=1073)	unclear	24W 1 year	Unclear	1) LVEF decrease ≥10 points (n=114) 2)CHF(n=7) 3) Cardiac death(n=0)
Pooja P. Advani	2015	USA	A+C→T(N=205)	49	9.2 year	Unclear	1) LVEF decrease ≥10 points (n=42) 2) LVEF decrease 15 ≥points (n=19) 3) LVEF decrease to below the LLN (n=13) 4) Cardiac death(n=2)
Patricia A. Ganz	2017	USA	A+C→T(N=220)	unclear	1) 18months(n=110) 2) 8.8 years (n=110)	Unclear	1) LVEF decrease ≥10% to <50% (n=3) 2) LVEF decrease ≥10% to <50%(n=5)
C. Hudis	1999	USA	A→T→C(N=42)	46	48 months	Metastatic	1) cardiac toxicities (n=0)
Roy E. Smith	2002	USA/Canada	A+C+T(N=89)	30-78	36.5months	Metastatic	1) LVEF decrease ≥20% (n=21) 2) CHF(n=3)
Edward H.Romond	2005	USA	A+C→T(N=625)	unclear	2 years	Non-metastatic	1) CHF(n=4) 2) Cardiac death(n=1)
Edward H. Romond	2012	USA	A+C→T(N=743)	49	7 years	Unclear	1) CHF(n=9) 2) Cardiac death(n=1)
Maysa M. Abu-Khalaf	2007	USA	A→T→C(N=85)	56.7	7 years	Metastatic	1) LVEF decrease <50% (n=7) 2) CHF(n=1) 3) Cardiac death(n=0)
Jean-marc A.Nabholtz	1997	USA	T→A→C(N=52)	49	2 months	Metastatic	CHF(n=1)
Elizabeth Tan-Chiu	2005	USA	A+C→T(N=814)	unclear	5 years	Non-metastatic	1) CHF(n=4) 2) Cardiac death(n=1)
J.M. Nabholtz	2001	France	T→A+C(N=40)	18-70	32 months	Metastatic	1) CHF(n=2)
D. Khayat	2001	France	A+C→T(N=44)	18-75	40.4 months	Metastatic	1) CHF(n=2)

## Data Availability

The data used to support the findings of this study are available from the corresponding author upon request.
